# Study on Baohe Pills Regulating Intestinal Microecology and Treating Diarrhea of High-Fat and High-Protein Diet Mice

**DOI:** 10.1155/2022/6891179

**Published:** 2022-05-17

**Authors:** KangXiao Guo, YongWang Yan, ChaoFeng Zeng, Ling Shen, YunShan He, ZhouJin Tan

**Affiliations:** ^1^Changsha Health Vocational College, Changsha, Hunan Province, China; ^2^Hunan University of Chinese Medicine, Changsha, Hunan Province., China

## Abstract

**Objective:**

To investigate the effects of Baohe pills on intestinal microorganisms and enzyme activities in mice with a high-fat and high-protein diet.

**Methods:**

45 KM male mice were randomly divided into the control group, the high-fat and high-protein diet group, and the Baohe pill intervention group. The mice in the high-fat and high-protein diet group and the Baohe pill intervention group were fed with the self-made high-fat and high-protein diet as the sole food source of the mice, and the mice in the control group were fed with the normal diet. Starting from the 7th day of the feed intervention, mice in the Baohe pill intervention group were given 0.28 g/mL of Baohe pill decoction twice a day at the dose of 6.67 g/(kg·day), each time of 0.35 mL for 6 days. Mice in the control group and the high-fat and high-protein diet group were given the same amount of distilled water by gavage. The general state of mice in each group was observed, and the changes of intestinal microorganisms and intestinal enzyme activities were analyzed by culturable microorganism technology and intestinal functional enzyme detection technology.

**Results:**

The excrement of mice fed with a high-fat and high-protein diet was relatively thin and wet, and the Baohe pill intervention could not improve the symptoms well. In the high-fat and high-protein diet group, the number of bacteria, *Escherichia coli*, *Lactobacillus*, and *Bifidobacterium*, was significantly lower than that in the control group (*P* < 0.01). Baohe pills could obviously increase the high-fat, high-protein diet for the number of culturable microorganisms in mice, the total number of bacteria, and the number of *Bifidobacteria* in the most significant (*P* < 0.01), but the number of bacteria, *Escherichia coli*, and the *Lactobacillus* are still significantly lower than the control group (*P* < 0.01). In terms of enzyme activity, both contents and mucosa, the Baohe pill could improve the activities of amylase, protease, sucrase, and lactase in high-fat and high-protein diet mice, which were significantly different from the control group (*P* < 0.05). In terms of microbial activity, the intestinal contents of high-fat and high-protein mice were lower than those of the control group, while the intestinal mucosa was higher than that of the control group, but the difference was not significant (*P* > 0.05). Baohe pills could improve the intestinal contents and intestinal mucosal microbial activity of mice, and the difference was significant in the high-fat and high-protein diet group (*P* < 0.05). *Discussion*. A high-fat and high-protein diet can destroy the physiological balance of the body, which is mainly reflected in the disturbance of intestinal flora and the decrease of some enzyme activities and microbial activity. Baohe pills can restore the number of intestinal flora to a certain extent and improve the activities of various digestive enzymes including protease and amylase.

## 1. Introduction

In recent years, the “three high” symptoms represented by hyperlipidemia have become an increasingly young disease. According to the statistics of the health department, since 2012, the overall prevalence of dyslipidemia in China has exceeded 40%, and the total detection rate of dyslipidemia among children and adolescents aged 6-17 is as high as 28.5% [1]. Unreasonable dietary structure is one of the main factors to induce dyslipidemia. Long-term excessive blood lipid level will cause hyperlipidemia, atherosclerosis diseases, and other cardiovascular and cerebrovascular diseases [2]. With the development of economy and the improvement of living standards, the food consumption structure has changed, which changed from a single mode of plant consumption to a multiple mode of animal and plant consumption. The nutritional demand pattern has also changed from a traditional food and vegetable-based carbohydrate and high fiber intake pattern to a new era of high fat, high sugar, high protein, and low fiber intake of grain and meat. Studies have shown that intestinal flora can promote the digestion and absorption of nutrients and play an important role in host energy metabolism and immune regulation. There are also associations between structural changes in the intestinal flora, dysfunction and obesity, and cardiovascular and cerebrovascular diseases [3–5]. Compared with western medicine treatment, TCM therapy can improve the structure composition of intestinal flora to balance gray energy supply and demand, which has the advantages of small side effects and strong safety and control.

Baohe pills come from the Tanxi Heart Law written by Zhu Zhenheng, including hawthorn, divine comedy, Pinellia, porkahoe, tangerine peel, forsythia, and radish seeds. The combination of medicine can play spleen and stomach, food, clearing heat, and clearing damp work. This compound reused hawthorn for the king medicine, the divine comedy, and radish son, and for the minister medicine, three drugs together can eliminate a variety of dietary stagnation. The pharmacological effect study shows hawthorn's many components have a lipid-lowering effect, such as hawthorn fruit gum five sugar, hawthorn flavonoids [6]. Hawthorn contains a variety of organic acids that can increase protease, pancreatic lipase, and other digestive enzyme activities and improve gastrointestinal movement. Turnip seed contains mustard base, linolenic acid, palmetto acid, oleic acid, and other components, which also have a certain effect on lowering blood lipid [7]. The research group fed mice with a high-fat and high-protein diet and intervened with the classic consumer agent Baohe pills. By analyzing the changes in cultured microbes and enzyme activity of the mouse intestinal tract, it provided an experimental basis for the application of Baohe pills in clinical practice and also provided suggestions for a reasonable diet during drug use.

## 2. Materials and Methods

### 2.1. Animals and Procedures

40 specific pathogen-free (SPF) Kunming mice were purchased from Hunan Slaccas Jingda Laboratory Animal Company with license number SCXK (Xiang) 2019-0004. All mice are male, with an average weight of about 20 ± 2 g. All procedures involving animals were reviewed and approved by the Animal Ethics and Welfare Committee of Hunan University of Chinese Medicine, animal license SCXK (Xiang) 2019-0009. Mice were reared in the Animal Experimental Center of Hunan University of Traditional Chinese Medicine in a clean and quiet environment with a temperature of 23-25°C and a humidity of 47-53%. After 2 days of adaptive feeding, 45 KM male mice were randomly divided into three groups, 15 mice per group: normal groups, high-fat, high-protein diet group, and Baohe pill intervention group. Among them, the high-fat, high-protein feed group and the Baohe pill intervention group used homemade special feed as the only source of experimental mice, and the normal group was fed the normal diet. After 6 days of the dietary intervention, the 7 d start Baohe pill intervention group was infused with 0.28 g/mL Baohe pill water infusion at a dose of 6.67 g/(kg day), twice a day at 0.35 mL. Equamount of distilled water was infused in normal and high-fat and high-protein feed groups for 6 days. The feed remains intact.

### 2.2. Medicine

Reference to literature and improve [8]. Hawthorn 18 g (Hebei), six divine comedy 6 g, Pinellia 9 g (Sichuan), Fuling 9 g (Hunan), tangerine 3 g (Zhejiang), forsythia 3 g (Shanxi), and raphani 3 g (Anhui) were all purchased in the First Affiliated Hospital of Hunan University of Chinese Medicine. In addition to the divine comedy, add the above medicinal materials into the porcelain pot with 500 mL, boil and then turn to low heat for 30 min, filter the residue and add 400 mL, continue to fry over low fire for half an hour, mix the mixture twice, and concentrate in a 76°C water bath pot to 150 mL. Divine comedy was developed into a fine powder with a mortar. After a 120 eye sieve, 6 g was added to the concentrated mixture and stirred well. Finally, it was diluted to 180 mL with distilled water to make a decoction solution with a concentration of 0.28 g/mL.

### 2.3. Reagents

High-fat, high-protein feed: milk powder from Nestle, bean powder from Huiyi, flour from Huiyi, meat floss from Anhui Lizhong at 1 : 2 : 1 : 1 mixed evenly, mix with appropriate water and paste, plastic with a syringe, dry in a 70°C oven for 72 h, shape close to ordinary maintenance feed. Reagents used in the determination of intestinal enzyme activities: Folin-phenol was purchased from Hefei Bomei Biotechnology Co. LTD. DNS reagent, O-nitrophenyl *β*-D-galactopyranoside (ONPG) reagent, and four substrate solutions were prepared in the lab. Acetone was purchased from Hunan Huihong Reagent Co. LTD (Hunan China). FDA was purchased from Shanghai Yuanye Biotechnology Co. LTD (Shanghai China), and sodium phosphate buffer was prepared in the lab [9].

### 2.4. Extraction of Intestinal Feces

All mice were sacrificed by cervical dislocation after being gavaged for treatment. The intestinal feces (from the jejunum to the rectum) of all mice in each group were collected, respectively, in a sterile environment and cooled in a 4°C refrigerator [10].

### 2.5. Intestinal Mucosa Extraction

Intestinal mucosa in each group was collected according to the collection method of sterile intestinal mucosa established by our research group. Under sterile conditions, the feces on the wall of the small intestine (the jejunum to the rectum) were washed with sterile saline, and then, the intestinal mucosa was scraped off using coverslips and cooled to -80°C liquid nitrogen tank.

### 2.6. Determination of Microbiota in Intestinal Feces

A certain amount of intestinal feces from each group were weighed aseptically and transferred into the corresponding group's triangle bottle filled with sterile water and glass beads. Triangle bottles were shaken on a bed temperature incubator at 120 rpm for 30 minutes to release microorganisms from intestinal feces completely. The number of microbiota was counted by dilution plate culture counting. The experiment was performed in triplicate. Bacteria were detected after being cultured in beef extract peptone AGAR medium at 37°C for 24 h; the number of *Lactobacillus* spp. and *Bifidobacteria* spp. was determined after being cultured, respectively, in MRS AGAR medium and BBL AGAR medium at 37°C for 48 h. Each dilution was repeated 3 times, and the average of each dilution was calculated to the number of bacteria per gram of intestinal feces.

### 2.7. Analysis of Enzyme Activities of Intestinal Mucosa in Mice

The intestinal mucosa sampled aseptically from each group was collected into the corresponding group's centrifuge tube filled with glass beads after being weighed. An appropriate amount of sterile water was then added. Bacteria suspensions of the intestinal feces of three groups were transferred from the triangle bottle into the corresponding group's centrifuge tube. Centrifuge tubes were shaken on a vortex mixer for 10 min to prepare crude enzyme of intestinal feces and mucosa. Then, crude enzymes were centrifuged at 3000 rpm for 8 minutes, and enzyme activities in the supernatant were analyzed by a UV spectrophotometer. Protease activity was determined by the Folin-phenol method; the activities of amylase and sucrase were determined by the DNS colorimeter method and lactase by the ONPG method. The unit of enzyme activity is defined according to the reference [11, 12].

### 2.8. Determination of Microbial Activity

The sample (intestinal mucosa and feces) was simultaneously added with 2.5 mL of FDA solution to sterile sodium phosphate buffer (final concentration, 10 *μ*g/mL), pH 7.6, and the mixture was incubated at 24°C on a rotary shaker. After 90 minutes, 2 mL of acetone was added to stop the reaction, and the value of A490 was determined. In addition, to set up a set of blank control groups, sterile water was used as a blank control. Three repeated tests were performed on each sample.

### 2.9. Statistical Analysis

Data were expressed as mean ± standard deviation (mean ± SD). Statistical analysis was performed by one-way ANOVA followed by Duncan's multiple range test using SPSS v23.0 (IBM Corp., Armonk, NY, USA). Differences between groups were considered statistically significant at *P* < 0.05.

## 3. Results

### 3.1. Fecal Status and Body Weight Changes in the Mice

By studying the fecal status and weight changes of the mice before and after the Baohe pill intervention, the normal group of mice showed black feces with certain hardness and shiny anal fur. Mice in the high-fat, high-protein diet and Baohe pill intervention groups were soft, brown, and sticky in the perianal and tail (Figure 1). All groups of mice gained weight at the end of the experiment. Body weight change and weight change rate were significantly lower in the Baohe pill intervention group than those in the normal mice (*t*_1_ = 2.653, *P*_1_ < 0.05; *t*_2_ = 2.202, *P*_2_ < 0.05). The high-fat, high-protein diet group was lower than the normal group, but not statistically different compared with the two groups (*P* > 0.05). Under the intervention, mice always had lower weight than the normal group and the high-fat, high-protein diet group, reflecting that bolus may have certain lipid-lowering effects (Table 1).

### 3.2. Effect of Baohe Pill on Diet and Water Intake in Mice with High-Fat and Protein Diet

As shown in Table 2 and Figures 2 and 3, mice with a high-fat and high-protein diet consumed significantly less food than mice on the normal diet (*P* < 0.05). After protection and bolus intervention, the food intake was significantly lower than that in the normal group (*P* < 0.05). In terms of drinking water, the high-fat, high-protein diet group had higher water than the Baohe pill intervention group than the normal group, but there was no statistical difference in daily water intake between the three groups (*P* > 0.05).

### 3.3. Effect of Baohe Pill on Organ Coefficient in Mice with High-Fat and Protein Diet

Organ coefficient is one of the main biological characteristics of experimental animals, which can be used to measure and reflect the functional state of animals, and is an item that must be observed and detected in drug safety evaluation [13]. The decrease in organ coefficient reflects organ atrophy and degenerative changes to a certain extent [14]. As can be seen from the following figure, a high-fat, high-protein feed can reduce the coefficients of the mouse liver, spleen, and thymus, but the difference was not statistically significant (*P* > 0.05). The recovery effect of Baohe pill intervention on the organ coefficient in mice with a high-fat diet was insignificant (*P* > 0.05) (Figure 4).

### 3.4. Effect of Baohe Pills on Gut Microbes in High-Fat, High-Protein Feed Mice

After high-fat and high-protein feed intervention, the total intestinal bacteria, *Lactobacillus*, and *Bifidobacteria* all decreased significantly compared with the normal group (total number of *t*_bacteria_ = 11.524, total *P*_bacteria_ < 0.01; *t*_E.coli_ = 10.040, *P*_E.coli_ < 0.01; *t*_Lactobacillus_ = 10.310, *P*_Lactobacillus_ < 0.01; *t*_*Bifidobacteria*_ = 5.435, *P*_Bifidobacterium_ < 0.01). Baohe pills increased the number of culturable microbes in the gut of mice with high-fat and high-protein diets, where the total number of bacteria and *Bifidobacteria* varied significantly compared with the high-fat, high-protein diet groups (total *t*_bacteria_ = −7.175, total *P*_bacteria_ < 0.01; *t*_Bifidobacteria_ = −7.840, *P*_Bifidobacteria_ < 0.01). In addition to *Bifidobacterium*, the total number of bacteria, *E. coli*, and *Lactobacillus* in the Baohe pill intervention group was significantly lower than that in the normal group (total number of *t*_bacteria_ = 8.670, total *P*_bacteria_ < 0.01; *t*_E.coli_ = 9.558, *P*_E.coli_ < 0.01; *t*_Lactobacillus_ = 6.401, *P*_Lactobacillus_ < 0.01) (Figure 5).

### 3.5. Effect of Baohe Pill on the Intestinal Mucosal Enzyme Activity of High-Fat, High-Protein Feed Mice

The integrity of intestinal mucosa is an important guarantee that intestinal digestive enzymes play the function of digestion and absorption of nutrients [15]. Many Chinese medicine chemicals can make the intestinal villi thicker, grow, and arrange more compact and orderly, thus having a significant impact on the generation and secretion of digestive enzymes [16, 17]. In other words, changes in enzymatic viability from the intestinal mucosa can reflect changes in the intestinal mucosal structure. From Table 3, the intestinal mucosal enzyme activity of mice with the high-fat, high-protein diet group was not statistically different compared with the normal group (*P* > 0.05), suggesting a less destructive effect of a short-term high-fat, high-protein diet on an intestinal mucosal structure. After treatment with Baohe pills, mouse mucosal protease, amylase, and sucrase were significantly higher than in the normal group (*t*_protease_ = −6.115, *P*_protease_ < 0.01; *t*_amylase_ = −14.531, *P*_amylase_ < 0.01; *t*_sucrase_ = −4.293, *P*_sucrase_ < 0.01; *t*_lactylase_ = −7.712, *P*_lactase_ < 0.01). In addition, the intestinal mucosal protease, amylase, and lactase activities were higher than in the high-fat and high-protein diet groups (*t*_protease_ = −6.854, *P*_protease_ < 0.01; *t*_amylase_ = −8.972, *P*_amylase_ < 0.01; *t*_lactase_ = −4.105, *P*_lactase_ < 0.01).

### 3.6. Effect of Baohe Pills on the Microbial Activity of High-Fat, High-Protein Feed Mice

Luciferin diacetic acid can be hydrolyzed by esterase, protease, and lipase [18], using FDA to reflect the changes of intestinal microbiota activity, microbiota, and intestinal enzyme activity [19]. From Figure 6, whether intestinal content or intestinal mucosa, the Baohe pill can significantly improve the microbial activity of high-fat and high-protein diet mice (*t*_content_ = −2.988, *P*_content_ < 0.05; *t*_mucosa_ = −9.387, *P*_mucosa_ < 0.01). The intestinal content of the high-fat and high-protein diet mice was less than normal, and the mucosal microorganism was higher than normal, but after statistical analysis (*P* > 0.05).

## 4. Discussion

### 4.1. Baohe Pills Can Treat High-Fat, High-Protein Diet Diarrhea by Regulating the Intestinal Flora

There is a large and complex microbial flora in the human body, which participates in human energy metabolism, growth and development, nutrient absorption, and many other processes and is closely related to a variety of diseases [20–22]. As can be seen from the above experimental results, the high-fat and high-protein diet can significantly reduce the total number of bacteria, *E. coli*, *Lacticate*, and *Bifidobobacteria* (*P* < 0.01) in normal mice, reflecting the damage of the mouse intestinal microecosystem, and the normal intestinal function is affected. The decreased activity of proteases and amylase in intestinal contents and intestinal mucosa can also reflect impaired normal intestinal function. *Lactobacillus* and *Bifidobacteria* are known probiotics in the mammalian gut. The membrane barrier formed by *Bifidobacteria* and intestinal epithelium suppresses the colonization and growth of pathogenic bacteria through occupation and competition to maintain human health; *Lactobacillus* can inhibit four intestinal pathogenic bacteria, *Escherichia coli*, *E. coli*, Salmonella, Shigella, and V. cholerae. After Baohe bolus intervention, the number of four culturable microbes increased, with the total number of bacteria and *Bifidobacterium*. The main chemical component in Baohe pills is organic acids, which can provide favorable conditions for the growth of probiotics such as *Bifidobacterium* and lactic acid bacteria. It has been found that Baohe pills can significantly increase the number of *Bifidobacterium*, Clostridium, Desulphururvibrio, and hydrogen-producing bacteria in the intestine of high-fat diet mice [23].

### 4.2. Baohe Pill Can Effectively Treat Diarrhea in Mice with High-Fat and High-Protein Diet by the Regulation of Intestinal Digestive Enzyme

Baohe pills can treat high-fat, high-protein diet diarrhea in region monogastric animals; the level of digestive enzyme activity in the intestinal tract reflects the strength of the body's digestive function to a certain extent. Changes in enzyme activity reflect the function of the small intestinal mucosa, but also the structural changes and activity changes of the flora in the gut [24]. Amylase and proteases are two important digestive enzymes in the gut. From the above experimental results, it can be found that in both the intestinal contents and the intestinal mucosa, Baohe pills can significantly improve the activity of protease and amylase in mice with a high-fat and high-protein diet. This experimental result basically agrees with the previously reported pharmacological effects of [25]. Intestinal digestive enzymes are divided into endogenous digestive enzymes and exogenous digestive enzymes according to their source. In the group of Baohe pills, the multiple drugs themselves contain amylase or protease, which can help the body digest and absorb protein and carbohydrates. For example, the Baohe pill hawthorn contains a certain amount of amylase but also contains pepsin agonist, which can increase pepsin activity [26]. Divine comedy is one of the widely used koji, fermented by Artemisia annua, grass, ear grass, bitter almond, polygonum, red beans, and flour. The pharmacodynamic basis of the divine comedy is mainly various enzymes (malt oligosanase, protease, amylase, etc.) and a variety of microbial metabolites (monosaccharides, oligosaccharides, and long-chain fatty acids), which is a commonly used clinical consumer drug [27]. The traditional method of traditional Chinese medicine is easy to destroy the enzymes and some beneficial microorganisms in the divine comedy, so in ancient times, the divine comedy into pills is directly administered [28]. In the experimental study of the divine comedy, the divine comedy is also often made into a suspension and used directly for gavic. In the course of this experiment, we used the traditional Chinese medicine decoction method into the decoction and grind the divine comedy into a fine powder and evenly disperse into the decoction. This move can fully guarantee that the pharmacodynamic substances of the divine comedy are not destroyed, and it is also an important reason for the improvement of protease and amylase in the Baohe pill intervention group, calculating the enzymatic activity of intestinal digestive enzymes.

## 5. Summary

The high-fat and high-protein diet can destroy the balance under the body's physiological conditions, mainly reflected in the intestinal flora disorder and the decline of some enzyme activity and microbial activity. The research group fed mice with a high-fat and high-protein diet and intervened with the classic consumer agent Baohe pill. The innovation of the research lies in the method of the gut microecology, analyzing the changes in cultured microbes and enzyme activity of the mouse intestinal tract; Baohe pill intervention can restore the amount of intestinal flora to some extent and improve the activity of various digestive enzymes, including protease and amylase. The study also confirmed the performance of a high-fat and high-protein diet that may have some inhibitory effect on protection and pill efficacy, suggesting that special attention should be paid to the diet during drug treatment. The results of these studies provided experimental basis for the application of Baohe pill in clinical practice, not only provided suggestions for a reasonable diet during drug use but also provided some experimental basis for the development of lipid-lowering products.

## Figures and Tables

**Figure 1:** Observation of the state of mouse feces. Note: normal group mice showed black feces with certain hardness and shiny anal fur. Mice in the high-fat, high-protein diet and Baohe pill intervention groups were soft, brown, and sticky in the perianal and tail.

**Figure 2:** Effect of Baohe pills on food intake in mice. Note: mice with a high-fat and high-protein diet consumed significantly less food than mice on the normal diet. After protection and bolus intervention, the food intake was significantly lower than that in normal group.

**Figure 3:** Effect of Baohe pills on water consumption in mice. Note: high-fat, high-protein diet had higher water than the Baohe pill intervention group than the normal group, but there was no statistical difference in daily water intake between the three groups.

**Figure 4:** Effect of Baohe pill on the organ coefficient in mice. Note: organ coefficient is one of the main biological characteristics of experimental animals, which can be used to measure and reflect the functional state of animals, and is an item that must be observed and detected in drug safety evaluation. The decrease in organ coefficient reflects organ atrophy and degenerative changes to a certain extent.

**Figure 5:** Effect of Baohe pills on the intestinal microbes of mice with high-fat and high-protein feed. After high-fat and high-protein feed intervention, the total intestinal bacteria, *Lactobacillus*, and *Bifidobacteria* all decreased significantly compared with the normal group. Baohe pills increased the number of culturable microbes in the gut of mice with high-fat and high-protein diets, where the total number of bacteria and *Bifidobacteria* varied significantly compared with the high-fat, high-protein diet groups.

**Figure 6:** Effect of Baohe pill on microbial activity in mice with a high-fat, high-protein diet. Note: compare with the normal group: a represents *P* < 0.01; A represents *P* < 0.05; compare with the model group: b represents *P* < 0.01; B represents *P* < 0.05.

**Table 1:** Effect of Baohe pill on body weight change and change rate in mice.

Group	Body weight change (g)	Weight change rate (%)
Normal group	3.89 ± 1.13	12.07 ± 3.75
High-fat, high-protein diet group	3.08 ± 1.49	10.14 ± 4.72
Baohe pill intervention group	2.38 ± 1.85^A^	7.94 ± 6.06^A^

Note: A represents comparison with the normal group, *P* < 0.05; B represents comparison with the high-fat, high-protein diet group, *P* < 0.05.

**Table 2:** Daily active food intake of mice in each group (g).

Group	The first day	The second day	The third day	The 4th day	The 5th day	The 6th day	The 7th day
Normal group	5.93	7.13	7.39	7.85	7.14	7.48	7.12
High-fat, high-protein diet group	4.53	5.66	4.69	4.57	4.85	5.26	5.07
Baohe pill intervention group	3.99	6.93	3.67	5.42	5.30	8.24	6.26

Note: autonomous daily feeding volume = daily feeding amount − daily feed surplus.

**Table 3:** Effect of Baohe pill on the intestinal mucosal enzyme activity of high-fat, high-protein feed mice (U/g).

Group	Protease	Amylase	Xylanase	Cellulase	Saccharase	Lactase
Normal group	0.34 ± 0.02	1.33 ± 0.02	0.60 ± 0.07	0.04 ± 0.01	1.82 ± 0.14	9.12 ± 0.22
High-fat, high-protein diet group	0.34 ± 0.02	1.60 ± 0.03	0.56 ± 0.04	0.03 ± 0.01	1.99 ± 0.10	10.08 ± 0.56
Baohe pill intervention group	0.41 ± 0.01^ab^	2.06 ± 0.08^ab^	0.71 ± 0.17	0.04 ± 0.01	2.19 ± 0.05^a^	12.15 ± 0.64^ab^

Note: comparison with the normal group: a represents *P* < 0.01; A represents *P* < 0.05; comparison with the model group: b represents *P* < 0.01; B represents *P* < 0.05.

## Data Availability

The datasets used and analyzed during the current study are available from the corresponding author on reasonable request.
